# Analysis of the Effect of Exercise Combined with Diet Intervention on Postoperative Quality of Life of Breast Cancer Patients

**DOI:** 10.1155/2022/4072832

**Published:** 2022-05-27

**Authors:** Lihua Lu, Xiaofeng Chen, Ping Lu, Jianli Wu, Yunxia Chen, Tiantian Ren, Yiju Li, Xiang Zhong

**Affiliations:** ^1^Thoracic and Breast Surgery, Affiliated Hospital of Nantong University, China; ^2^School of Nursing, Medical College, Nantong University, China

## Abstract

To analyze the effect of exercise combined with diet intervention on postoperative quality of life of breast cancer patients, a total of 104 breast cancer patients randomly selected from October 2019 to September 2020 who received systemic adjuvant endocrine drug therapy in our hospital for the first time were divided into the observation group and control group as the research subjects. The control group was given exercise and exercise intervention on the basis of routine nursing, and the observation group was given exercise and exercise combined with diet intervention on the basis of basic nursing. Nutritional indexes, anxiety and depression, sleep quality, cancer-induced fatigue, and life quality were observed in both groups. The nutritional indicators of the observation group were slightly different from the control group after exercise and diet intervention, indicating that the observation group's data was higher than the control group (*P* > 0.05). The HAMA (human anti-mouse antibody) and HAMD (Hamilton depression scale) ratings of the two groups did not differ significantly (*P* > 0.05). Both groups' HAMA and HAMD ratings improved after intervention; although, the control group's increase was bigger than the observation group (*P* < 0.05). Both groups' poor sleep quality assessment (PSQI) scores improved after intervention, with the observation group's increase rate being lower than the control group (*P* < 0.05); the control group's sleep time fell more than the observation group (*P* < 0.05).

## 1. Introduction

The World Health Organization (WHO) pointed out that breast cancer has become the highest incidence of malignant tumors in women worldwide [1]. Compared with other countries, the incidence of breast cancer in China is at a low level. However, the prevalence of breast cancer in China has been steadily increasing in recent years [2, 3]. The main treatment for breast cancer is surgical treatment, and in addition to radiotherapy and chemotherapy after surgery, the estrogen receptor and/or progesterone receptor positive patients need to receive at least 5 years of endocrine therapy [4]. Studies have shown that the 5-year survival rate of Chinese breast cancer patients can exceed 88%, which has become a kind of malignant tumor with a relatively optimistic prognosis [5, 6]. But as patients live longer, other related problems emerge [7]. As a result of the adverse reactions caused by the disease and the treatment process, a variety of physical and psychological problems are exposed, such as the appearance of negative emotions, poor sleep quality, and cancer-related fatigue [8]. How to reduce the impact of these negative behaviors on patients and improve the quality of life of patients after surgery has become the focus of medical research [9, 10]. In this study, data of 104 cases of breast cancer patients treated in our hospital were analyzed to explore the influence of exercise combined with diet on postoperative quality of life of breast cancer patients, and the results are reported as follows.

The arrangements of the paper are as follows:

Section 2 discusses the materials and methods.  Section 3 analyzes the result.  Section 4 examines the various discussions.  Section 5 concludes the article.

## 2. Materials and Methods

### 2.1. General Information

A total of 104 breast cancer patients who received the first systemic adjuvant endocrine drug therapy in our hospital from October 2019 to September 2020 were enrolled by convenience sampling. Patients signed informed consent before grouping, and this study had been approved by the ethics committee of our hospital.

#### 2.1.1. Inclusion Criteria

The inclusion criteria were as follows: **①** diagnosed by pathology as primary breast cancer with stage I ~ A and underwent surgical treatment in our hospital, **②** after receiving chemotherapy in our hospital, the survival time was more than 6 months, **③** the body was free of serious comorbidities that could affect the results, and **④** sane and able to communicate normally.

#### 2.1.2. Exclusion Criteria

The exclusion criteria were as follows: **①** patients or their family members refused to accept the intervention in this study, **②** patients who had been exercising regularly before, **③** accompanied by other diseases that affect the patient's activities, **④** had mental disorders and was unable to communicate, and **⑤** life expectancy was less than 1 year.

Patients were divided into the control group (*n* = 52) and observation group (*n* = 52) according to the random number table method. There was no significant difference in general clinical data between the two groups (*P* > 0.05).General information was shown in Table 1.

### 2.2. Methods

#### 2.2.1. Conventional Nursing

During their stay, all patients received normal treatment, which included exposing them to the hospital environment and staff following admission in order to help them transition into their roles as quickly as possible. Help patients to complete the examination, assist them to complete the nursing operation, eliminate the patient's tension and fear of psychology, and ensure the treatment of cooperation.

#### 2.2.2. Nursing of the Control Group

Exercise was administered as follows, based on traditional nursing: the nursing team will construct the appropriate exercise strategy based on the unique features of the patients. Exercise 3 times a week for the first three weeks for about 15 minutes and then gradually increase: maximum heart rate = 220 − patient age. During weeks 1 to 6, the intensity of exercise was 50% of the maximum heart rate. The intensity of exercise was 60% of maximal heart rate for weeks 7 to 10. All patients should choose an exercise that includes three parts: warm-up exercise, genuine exercise, and rest and relaxation, with a time control ratio of 1 : 3 : 1. Regular health education was taken for patients, to teach patients the benefits of physical exercise for breast cancer recovery.

#### 2.2.3. Nursing of the Experimental Group

On the basis of exercise nursing in the control group, diet nursing intervention measures were given, as follows: **①** diet nursing intervention on admission: to understand the eating habits and nutritional status of patients after admission and inform family members and patients of dietary taboo information, **②** dietary intervention during chemotherapy: nursing staff should guide patients to eat high protein, high energy, high vitamin, and other diets and advice patients to eat a high-fiber diet, and **③** dietary care after discharge: develop a targeted diet plan, diet, and nutrition manual for patients upon discharge.

### 2.3. Observational Index

Observational index included the following:

1. Nutritional indicators: hemoglobin, serum albumin, lymphocyte count, and body mass index
2. Anxiety and depression: the Hamilton Anxiety Scale (HAMA) was used to score patients' anxiety [11]. The higher the anxiety level, the higher the score. The Hamilton Depression Scale (HAMD) was used to score the patients' depression [12]. The higher the score, the more depressed
3. Sleep quality: the Pittsburgh Sleep Quality Index (PSQI) was used to score patients' sleep quality. The scores were added up to a total score, which ranged from 0 to 21, with higher scores indicating poorer sleep quality
4. Cancer-related fatigue: the Piper fatigue scale was used to evaluate patients' cancer-induced fatigue [13]. Each item was scored on a scale of 0 to 6, with higher scores indicating more severe cancer-related fatigue
5. Quality of life: quality of life was assessed using the Concise Health Status Questionnaire (SF-36) and the Inventory Scale (QLQ-C30). The higher the score, better the quality of life

### 2.4. Statistical Method

SPSS 17.0 Chinese version was used for data input and data processing. Measurement data was expressed as (*x* ± *s*). Independent sample *t*-test was used for analysis. Counting data is expressed as a percentage, *χ*^2^ test was used for analysis, and *P* < 0.05 was considered statistically significant.

## 3. Results

### 3.1. Results of Nutritional Index

After exercise and diet intervention, there was a slight difference in the nutritional indexes of the observation group compared with the control group, that was the data of the observation group was higher than that of the control group (*P* < 0.05). Results of nutritional index were shown in Table 2.

### 3.2. Results of Anxiety and Depression

The two groups' HAMA and HAMD scores were compared before and after intervention. Before intervention, there was no significant difference between the two groups' HAMA and HAMD scores (*P* > 0.05). After intervention, HAMA and HAMD scores in both groups were increased, and the increase in the control group was greater than that in the observation group (*P* < 0.05). Results of anxiety and depression were shown in Table 3.

### 3.3. Results of Sleep Quality

After intervention, the PSQI scores of both groups were improved, and the increase rate of observation group was less than that of the control group (*P* < 0.05); the sleep time in the control group decreased more than that in the observation group (*P* < 0.05). Results of sleep quality were shown in Table 4.

### 3.4. Results of Cancer-Induced Fatigue

Comparison of cancer-induced fatigue scores between the two groups before and after intervention showed that after the intervention, the scores of all dimensions of cancer-induced fatigue were increased in both groups, and the increase rate in the control group was higher than that in the observation group (*P* < 0.05). Results of cancer-induced fatigue were shown in Table 5.

### 3.5. Results of Quality of Life

After treatment, the quality of life scores in both groups increased, and the increase rate in the control group was less than that in the observation group (*P* < 0.05). Results of quality of life were shown in Table 6.

## 4. Discussion

Breast cancer is a frequent disease in clinical practice, and its frequency is rising year after year, posing a major threat to patients' physical and mental health [14, 15]. Some researchers have discovered that eating patterns, radioactive chemicals, living routines, genetics, and other variables are all linked to disease [16]. Exercise can obviously improve the blood circulation of the body, promote the metabolism of the tissue, improve the body function, and provide sufficient guarantee for the operation of other systems of the body. Continued exercise can also stimulate the body's pituitary gland to secret endorphins, improve the central nervous system response ability, and increase the body's tolerance to stimulation [17, 18]. The human body in the movement of the nervous system will appear weak electrical stimulation, and this stimulation can relieve muscle tension and mental depression and relax the cortex of the brain, so that the degree of psychological tension is weakened [19]. Due to the differences between the constitutions of patients, it is easy to cause different degrees of adverse reactions, such as loss of appetite, nausea, and vomiting, which will seriously affect the intake of nutrients, induce malnutrition, and other complications, and further reduce the resistance, thus affecting the effect of chemotherapy [14, 20].

This study showed that after exercise and diet intervention, there was a slight difference in the nutritional indexes of the observation group compared with the control group, that was the data of the observation group was higher than that of the control group (*P* < 0.05). HAMA and HAMD scores of the two groups had no significant difference (*P* > 0.05). After intervention, HAMA and HAMD scores in both groups were increased, and the increase in the control group was greater than that in the observation group (*P* < 0.05). Both groups' PSQI scores improved after intervention, but the observation group's increase rate was lower than the control group (*P* < 0.05); the control group's sleep time fell more than the observation group (*P* < 0.05). The scores of all dimensions of cancer-induced weariness increased in both groups after the intervention, with the increase rate in the control group being larger than the observation group (*P* < 0.05).

## 5. Conclusion

The human body in the movement of the nervous system will appear weak electrical stimulation, and this stimulation can relieve muscle tension and mental depression and relax the cortex of the brain. Exercise combined with diet intervention in breast cancer patients can alleviate the negative emotions of patients, reduce the degree of cancer-related fatigue, and improve sleep and quality of life, which is worthy of application and promotion.

## Figures and Tables

**Table 1:** General information.

Projects		Observation group	Control group	*X* ^2^	*P*
Age		52.25 ± 12.30	54.12 ± 10.25	0.06	>0.05
Marriage	In marriage	41	39	0.04	>0.05
	Not in marriage	11	13		
Work	Yes	12	9	1.80	>0.05
	No	40	43		
Health care costs	Self-paying	3	4	0.02	>0.05
	Health care	49	48		
Mastectomy	Yes	38	37	0.12	>0.05
	No	14	15		
Lymph node metastasis	Yes	8	9	0.08	>0.05
	No	44	43		
Maximum tumor diameter		2.04 ± 1.14	1.85 ± 1.09	0.25	>0.05

**Table 2:** Results of nutritional index.

Groups	Cases	Serum albumin (g/L)	Hemoglobin (g/L)	Body mass index (kg/m^2^)	Lymphocyte count (×10^9^/L)
Observation group	52	36.45 ± 2.63	119.44 ± 3.55	20.24 ± 1.89	1.45 ± 0.65
Control group	52	25.01 ± 1.04	102.14 ± 1.57	15.87 ± 1.02	0.21 ± 0.27

**Table 3:** Results of anxiety and depression.

Groups	Cases	Time	HAMA	HAMD
Observation group	52	Before intervention	12.65 ± 2.01	14.78 ± 2.44
		After intervention	14.14 ± 3.02	17.34 ± 3.01
Control group	52	Before intervention	12.57 ± 2.08	15.14 ± 2.12
		After intervention	16.52 ± 3.21	20.58 ± 2.62

**Table 4:** Results of sleep quality.

Groups	Cases	Time	PSQI	Sleep time (h)
Observation group	52	Before intervention	10.55 ± 3.01	7.78 ± 2.04
		After intervention	12.13 ± 2.04	6.46 ± 0.84
Control group	52	Before intervention	10.14 ± 2.17	7.82 ± 1.64
		After intervention	14.64 ± 3.12	5.67 ± 0.41

**Table 5:** Results of cancer-induced fatigue.

Groups		Observation group (*n* = 52)	Control group (*n* = 52)
Behavior	Before intervention	4.160 ± 0.712	4.133 ± 0.855
	After intervention	4.753 ± 0.271	5.611 ± 0.170
Feeling	Before intervention	4.122 ± 0.444	4.133 ± 0.511
	After intervention	4.351 ± 0.313	5.360 ± 0.482
Emotion	Before intervention	4.052 ± 0.343	4.061 ± 0.522
	After intervention	4.341 ± 0.255	5.255 ± 0.655
Cognition and mood	Before intervention	4.042 ± 0.383	4.022 ± 0.444
	After intervention	4.521 ± 0.272	5.133 ± 0.344
Overall assessment	Before intervention	4.050 ± 0.652	4.011 ± 0.780
	After intervention	4.741 ± 0.322	5.322 ± 1.022

**Table 6:** Results of quality of life.

Groups	Cases	Time	SF-36	QLQ-C30
Observation group	52	Before intervention	58.455 ± 4.061	59.460 ± 6.744
		After intervention	69.580 ± 3.662	74.522 ± 7.455
Control group	52	Before intervention	57.721 ± 4.062	58.044 ± 7.133
		After intervention	63.581 ± 4.070	70.311 ± 2.544

## Data Availability

The data used to support the findings of this study are included within the article.
